RETRACTED

# Sports Injury Modeling of the Anterior Cruciate Ligament Based on the Intelligent Finite Element Algorithm

**DOI:** 10.1155/2021/3606863

**Published:** 2021-12-09

**Authors:** Xia Huang

**Affiliations:** Institute of Physical Education, Jianghan University, Hubei 430056, China

## Abstract

In order to solve the problem of sports injury modeling of the anterior cruciate ligament, a method based on the intelligent finite element algorithm is proposed. Considering the transverse isotropy of the ligament, this paper constructs a 3D finite element model of the knee joint based on medical image data. The same ligament constitutive equation was used to fit the parameters of stress-strain mechanical experimental curves of three different anterior cruciate ligaments, and the effects of different anterior cruciate ligament mechanical parameters on kinematics and biomechanical properties of the knee joint were compared. The experimental results show that, in models 1, 2, and 3, the maximum stress values appear in the posterolateral of the femoral attachment area of the ligament, which are 16.24 MPa, 16.36 MPa, and 22.05 MPa, respectively. However, the stress values at the tibial attachment area are 9.80, 13.8, and 13.93 MPa, respectively, and the stress values at the anterolateral part of the middle ligament are 6.36, 11.89, and 12.26 MPa, respectively, which are all smaller than those at the femoral attachment area, which also quantitatively explains the clinical phenomenon that ACL fracture often occurs in the femoral attachment area in practice. Thus, the three-dimensional finite element model of the knee joint highly simulates the structure and material properties of the knee joint. This method proves that the intelligent finite element algorithm can effectively solve the modeling problem of sports injury of the anterior cruciate ligament.

## 1. Introduction

Knee joint is not only because of its complex structure but also because of its complex biomechanical properties. As the largest and most complex joint of the human body, knee joint is located between the hip joint and ankle joint, and it is the hub of lower limb activities. More and more people are aware of its importance and related diseases, and their research is getting deeper and deeper. According to the analysis of 2725 cases of sports injuries in various sports events by the Institute of Sports Medicine, knee injuries accounted for 25.82%, accounting for the first of all sports injuries [1]. Different types and degrees of knee injuries have seriously affected athletes' training and sports performance. Therefore, in order to make better prevention and rehabilitation plans or provide a scientific basis for researchers, it is necessary to study its pathogenesis. Knee joint is not only because of its complex structure but also because of its complex biomechanical properties. The anatomical structure, mechanical environment, and functional requirements of the knee joint make it one of the most frequently damaged joints [2]. With the further improvement of people's understanding of the importance of knee joint injury, people pay more and more attention to the study of biomechanical properties of the knee joint. The traditional experimental method of isolated specimens has contributed to the biomechanical study of the anterior cruciate ligament, but there are still many defects, such as some physiological and pathological conditions are difficult to simulate, and the stress measurement is not accurate enough. The finite element analysis method has incomparable advantages over the in vitro specimen experiment and effectively makes up for the deficiency of the in vitro experiment [3].

RETRACTED

In recent years, many scholars have put forward biomechanical models of different knee joints and made some research progress. Huang et al. made extensive and in-depth research on the causes of bone tunnel enlargement. However, due to the limitations of in vitro specimen experiments, many difficulties have arisen in the research. Finite element analysis is an important mechanical calculation method. In recent years, the biomechanical research and application of ACL reconstruction has developed rapidly, which is a good supplement to the in vitro specimen experiment. The finite element model of the knee joint mainly includes the tibia, femur, articular cartilage, and meniscus, but there is no ligament model around the knee joint. However, ligament is an important stabilizing device of the knee joint, which is indispensable for biomechanical research of the knee joint [4]. Zeng et al. believed that the knee joint model established by Zeng et al. includes the ligaments around the knee joint and the tibial and femoral tunnels used for ACL reconstruction, which provides a valuable tool for biomechanical study of ACL reconstruction [5]. Xu et al. obtained the mechanical curves of ligaments in vitro and fitted the parameters, directly using the mechanical models and parameter settings in other literature studies [6]. Biomechanical models of different knee joints have been proposed, and some progress has been made. However, due to the complexity of the anatomical structure, material properties, movement forms, and load distribution of each component of the knee joint, people cannot accurately describe various properties and behaviors of the knee joint at present. With the rapid development of modern computer technology and the gradual improvement of finite element software, finite element analysis is gradually attracting people's attention. Finite element analysis of the knee joint has become the focus of biomechanical research of the knee joint [7]. The three-dimensional finite element model of the knee was established by using CT images of healthy human knee joints, and the biomechanical properties of the anterior cruciate ligament, posterior cruciate ligament, medial collateral ligament, and lateral collateral ligament of the knee joint were analyzed when the knee calves were varus, and the tibia was subjected to different forward and backward forces. It reveals the biomechanical characteristics of knee joint movement comprehensively and provides a theoretical basis for sports training and analysis and prevention of knee joint movement injury.

RETRACTED

## 2. Research Methods

### 2.1. Model Establishment

The left knee joint of a healthy woman (36 years old) was scanned by magnetic resonance imaging in sagittal and transverse directions, which were used to obtain the geometric contour information of the main ligaments, bones, menisci, and other tissues of the knee joint. The scanning layer was 2 mm thick, the spacing was 0 mm, and the resolution was 0.371 mm/pixel (the field of view was 190 mm, and the pixel matrix was 512 × 512). Scanning conditions were as follows: selected bone tissue window, layer spacing 2 mm, a total of 113 layers, and scanning data directly stored according to DICOM 3.0 standard.

The obtained medical images are saved in the DICOM format, and the 3D knee joint model is reconstructed by importing 3D reconstruction software Mimics 13.1 (Materialise, Belgium). The model includes the main tissues of the knee joint: femur, tibia, cartilage, meniscus, anterior cruciate ligament, posterior cruciate ligament, medial collateral ligament, and lateral collateral ligament. The reconstructed three-dimensional knee joint model was introduced into finite element software ABAQUS 6.10 (Dassault Systemes Simulation Company, USA) to divide the second-order tetrahedron element, and the three-dimensional finite element model of the knee joint was obtained [8].

### 2.2. Establishment of the Finite Element Model of the Knee Joint and Tibia-Femur Tunnel

The solid model IGES file generated from Geomagic is imported into finite element analysis software ANSYS 9.0 (ANSYS Company, USA), and each solid structure is meshed with second-order tetrahedral elements. The proximal tibia and fibula adopt a rod unit only bearing pressure, and other tissue contact parts such as “cartilage-cartilage” and “cartilage-meniscus” adopt a frictionless contact setting. The material parameters are shown in Table 1. In order to perform 3D visualization of the CT data, medical image processing software IMICS was used to read DICOM grid data directly, the gray value of the bone and ilium in the images was extracted, and the gray value range of threshold was adjusted. The bone is separated from its surrounding tissue, the image with the gray value in the selected range is automatically marked, and the bone contour line of each layer is generated. The cartilage NURBS surface is divided into three-dimensional 8-node structural shell elements, and the self-adaptive closed-shell structure is connected to each bone tissue model. The ligament tissue simulated by the three-dimensional tension-only element includes the posterior cruciate ligament, medial and lateral collateral ligament, and patellar ligament, and the nonlinear elastic material is set, and the initial cross-sectional area is selected [9].

RETRACTED

The tibial-femoral tunnel used for ACL reconstruction was obtained by the Boolean operation of 7.5 mm diameter through the cylinder and tibial solid model. The solid model of the tibia and femur with the tunnel is meshed with the SOLID92 element. The isometric point of the tibial tunnel is located in front of the intercondylar spine on the medial side of the tibial plateau, 7 mm ahead of the stop point of the posterior cruciate ligament, and the tunnel forms an angle of 30 with the longitudinal axis of the tibia on the coronal plane. The sagittal plane is at 65 with the tibial plateau plane. The equal-length point of the femur is located in the lateral wall of the intercondylar fossa, 6 mm in front of the apex. The coronal tunnel is 30 with the long axis of the femur, and the sagittal tunnel is 25 with the long axis of the femur [10].

### 2.3. Material Properties

In this study, the density, elastic modulus, and Poisson's ratio of different materials were calculated according to different gray values of CT scan images, and the assignment problem of bone tissue with nonuniform material properties and anisotropic mechanical properties was realized. Assuming that the femur and tibia are homogeneous and isotropic linear elastic materials, elastic modulus *E*=14.22 GPa and Poisson's ratio *v*=0.3. The simple pendulum period of human walking is l second, which is far less than the viscoelastic effect time of cartilage. Therefore, the viscoelasticity of cartilage can be ignored in this study, which is defined as homogeneous isotropic linear elastic material. *E*=5 MPa and *v*=0.46. The material properties of the meniscus can be obtained: *E*=59 MPa and *v*=0.49 [11].

The fibers with similar orientation are distributed in the matrix composed of water, proteoglycan, and glycolipid, which constitute the fiber composite structure of the ligament. For the description of the mechanical properties of the ligament, this paper assumes that it is transversely isotropic superelastic material and adopts the constitutive equation of strain energy function. The strain energy equation of the ligament is divided into the volume part which describes the volume change, *ψ*_*vol*_, and the offset part describing the shape change, *ψ*_*iso*_, in which the offset part can be divided into matrix part $\psi_{\text{iso}}^{m}\left(\bar{C}\right)$ and fiber portions *ψ*_iso_^*f*^(*λ*).

RETRACTED

The strain energy formula is as follows:

(1) $$\begin{array}{c} \psi =\psi_{\text{vol}}\left(J\right)+\psi_{\text{iso}}^{m}\left(\bar{C}\right)+\psi_{\text{iso}}^{f}\left(\lambda \right). \end{array}$$

Type: *J* is the deformation gradient tensor. *F* Jacques ratio of $\bar{C}$ is Cauchy–Green deformation gradient tensor $\left(\bar{C}=J^{-2/3}C\right)$. Extensibility $\left(\bar{\lambda }\right)$ can be calculated by the deformation of materials and the initial direction of fibers (*a*_0_). It can be calculated as $\left({\bar{\lambda }}^{2}=a_{0}\cdot \bar{C}\cdot a_{0}\right)$ by assuming that the center of the attachment area at both ends of the ligament is the initial fiber direction of the ligament. According to the quasi-incompressibility of the ligament, its mass can be defined by penalty function:

(2) $$\begin{array}{c} \psi_{vol}\left(J\right)=\frac{1}{2\;D}\ln\;J^{2}. \end{array}$$

The deflection of the strain energy function of the matrix is assumed to be a neo-Hookean superelastic model, and the formula is

(3) $$\begin{array}{c} \psi_{\text{is}o}^{m}\left(\bar{C}\right)=C_{1}\left({\bar{I}}_{1}-3\right), \end{array}$$

where *C*_1_ is the coefficient of the neo-Hookean model. *D* is the reciprocal of bulk modulus, which can be calculated by formula *D*=(1/2000*C*_1_).

Because collagen fibers in ligaments can hardly bear ballast, the deviation of the strain energy function of fibers can be defined as

(4) $$\begin{array}{c} \bar{\lambda }\frac{\partial \psi_{\text{iso}}^{f}}{\partial \bar{\lambda }}=0\left(\bar{\lambda }<1\right),\\ \bar{\lambda }\frac{\partial \psi_{\text{iso}}^{f}}{\partial \bar{\lambda }}=C_{3}\left(e^{c_{4}\left(\bar{\lambda }-1\right)}-1\right),\;1\leq \bar{\lambda }\leq \lambda^{*},\\ \bar{\lambda }\frac{\partial \psi_{\text{iso}}^{f}}{\partial \bar{\lambda }}=C_{5}\bar{\lambda }+C_{6},\;\bar{\lambda }>\lambda^{*}, \end{array}$$

where *λ*^*∗*^ is the elongation when the fiber is straightened, that is, the inflection points between the exponential segment and the straight segment in the stress-strain curve.

RETRACTED

In order to study the influence of the change of the mechanical properties of the anterior cruciate ligament on the simulation results of the knee joint, 3 finite element models of the knee joint with different ACL mechanical properties were constructed in this paper. As shown in Figure 1, the mechanical experimental curves of the ACL in models 1, 2, and 3 are taken from the literature method. Based on these three different experimental data of ligament mechanics, the mechanical constitutive equation constructed by Bin et al. was fitted with parameters. Three groups of different material parameters were obtained for the finite element analysis of the knee joint. The material parameters of other ligaments are available, as shown in Table 2 [12].

## 3. Experimental Results

ACL starts from the medial side of the lateral condyle of the femur and ends in front of the intercondylar crest of the tibia in the anteroposterior and medial directions, which mainly limits the backward movement of the femur or the forward movement of the tibia. In order to analyze the influence of ACL mechanical properties on the whole displacement of the knee joint and the stress distribution of intra-articular tissues, according to the existing ACL mechanical property curves, this paper constructs three-dimensional finite element models of the knee joint with three different ACL properties. The finite element simulation results of the knee joint under 134 N femoral backward thrust load are obtained. According to the boundary conditions of the model, the three translation displacement values of the knee joint are taken from the femur, that is, the midpoint of the axis of the femoral epicondyle. Two rotational displacement values were taken from the tibia [13]. The rotation angles of LCL and MCL tibial attachment points relative to tibial plateau reference points were averaged to obtain the corresponding rotation displacement values. Under the same external load, the simulation results of the model are similar to the joint displacement values obtained from many previous knee biomechanical studies, which verifies the effectiveness of the finite element model of the knee joint in this paper. The 6-DOF displacement measuring manipulator system was used to measure the displacement of the knee joint of cadavers. It is found that the displacement of the joint in front and back, far and near, and inside and outside directions is 4.30 mm, 0.62 mm, and 0.39 mm, respectively, and the inward and outward rotation angles were 0.09° and 1.9°, respectively. Similar joint displacements (AP displacement is 4.0 mm, PD displacement is 0.3 mm, ML displacement is 0.6 mm, VV angle is 0.2°, and EI angle is 1.7) were measured by this system. In the retired experimental research, under the same load, the displacement of the knee joint in the AP direction is 3.5 mm and 4.16 mm, respectively [14]. These results indicate that the PCL is the primary structure to resist tibial anterior displacement during knee flexion, and the stress is mainly concentrated at the proximal tibial insertion, which is consistent with the clinical occurrence of PCL fracture at the insertion of the femur.

RETRACTED

## 4. Discussion

The simulated displacement results of the knee joint in this paper are different from the biomechanical experimental results of other researchers, which may be caused by the great differences among individuals. The displacement of the knee joint will be affected by the geometric size and mechanical properties of different joint tissues. First of all, the model in this paper is based on the medical image of a healthy Chinese adult woman's knee joint. The geometric size of joint tissue will be different from the samples in other experimental studies. Secondly, the mechanical properties of the ACL and other ligament tissues in this paper are taken from different mechanical experimental curves, which may be different from other experimental samples. It will also cause the difference between the simulation results and other experimental results [15]. Although the results are different, the simulation results in this paper are consistent with the whole displacement of the knee joint in the experiment, with little difference in the numerical value. Especially, the main displacement values (fore and aft displacement) of the knee joint under the backward thrust load of the femur are basically the same, which verifies the validity of the finite element model of the knee joint. Moreover, with the further development of material science, finite element analysis theory, and computer science, three-dimensional finite element model of the knee joint will become the main method for biomechanical analysis of the knee joint.

Table 3 lists the overall displacement of joints under three ACL mechanical properties. It can be seen that the kinematic performance of joint model simulation will be greatly affected by applying different ACL mechanical performance settings. Under the backward thrust of the femur of 134 N, the large displacement of the knee joint occurred in AP and ML directions, while the displacement in other directions was relatively small. EI displacement angle of joints is much larger than VV angle. In the relatively large three-degree-of-freedom movement of the joint (anteroposterior translation and anteroposterior rotation), the proximal displacement of the femur and medial rotation of the tibia in the three models are not much different, while the posterior displacement of the femur in the three models is quite different. On the contrary, this verifies the clinical viewpoint that the ACL mainly limits the anterior and posterior displacement of joints [16].

RETRACTED

In the comparative analysis of the influence of mechanical properties of the ACL on stress distribution in joint tissues, it can be found that the stress distribution trend on the ACL has little change, but the stress level has great change. As a relatively new biomechanical research method, finite element analysis has been gradually applied to the field of life science. It is a theoretical analysis, but it is difficult to obtain an accurate analytical solution due to the geometry, material properties, and irregular external loads of the knee joint. The Mises stress distribution in the ACL under three kinds of mechanical curves is shown. The stress on the ACL is mainly distributed in the posterolateral of femoral attachment area, posterolateral of tibial attachment area, and anterolateral of the ligament. Although the mechanical properties of ACLs have changed, the stress distribution trends on ACLs are basically the same [17]. In models 1, 2, and 3, the maximum stress values appeared in the posterolateral area of the femoral attachment of the ligament, which were 16.24 MPa, 16.36 MPa, and 22.05 MPa, respectively. However, the stress values at the tibial attachment area are 9.80, 13.8, and 13.93 MPa, respectively, and the stress values at the anterolateral part of the middle ligament are 6.36, 11.89, and 12.26 MPa, respectively, which are all smaller than those at the femoral attachment area, and the validity and reliability of the model are verified again, which also quantitatively explains the clinical phenomenon that ACL fracture often occurs in the femoral attachment area in practice. For other joint tissues, such as the MCL, meniscus, and cartilage, the stress distribution and magnitude of the ACL are basically the same, which indicates that the change of mechanical properties of the ACL has little influence on other joint tissues. A similar situation can be found in the strain distribution of joint tissues; that is, the strain distribution trend on the ACL has little change, but the strain level has great change, which shows the distribution of the maximum principal strain of the ACL under three kinds of mechanical curves. Similar to the stress distribution on the ACL, the maximum principal strain on the ACL is mainly distributed in the posterolateral of femoral attachment area, posterolateral of tibial attachment area, and anterolateral of the ligament, and the distribution trend is basically the same. In models 1, 2, and 3, the maximum principal strain of the posterolateral femur attachment area is 0.44, 0.24, and 0.20, respectively, while the maximum principal strain at the tibial attachment area is 0.35, 0.26, and 0.19, respectively, and the maximum principal strain at the anterolateral part of the middle ligament is 0.18, 0.15, and 0.12, respectively, which are all smaller than the principal strain at the femoral attachment area [18].

RETRACTED

In the traditional modeling method, articular cartilage is obtained by dividing solid elements between two hard bones. In the biomechanical modeling of the ankle in this model, Niu et al. first proposed the concept of adaptive closed-shell structure and applied it to plantar soft tissue modeling, which skillfully solved many problems existing in the field of finite element modeling of biological tissues. Because the thickness of knee cartilage is limited, its thickness is much smaller than that of other dimensions, so the application of solid element division will inevitably produce a large number of deformed elements, resulting in large calculation errors. The original image in the DICOM format obtained by CT scanning is preprocessed in Mimics without any format conversion, which avoids the loss of information, saves a lot of time, and reduces the workload. The definition of threshold 0 is used to complete the extraction of bone contour and realize automation. And the modeling speed and accuracy are improved. The effective solution before is to use entity units whose dimensions in one dimension of a single layer are much smaller than those in the other two dimensions for division. The thickness of cartilage in different positions was simulated by the size of the unit. This method is similar to the shell element in essence, but it is technically difficult to realize the simulation of tissue thickness by controlling the size of the solid element. In addition, the nodes on the edge have no adaptive function. In this model, the shell element is used to simulate the geometric features of cartilage, so as to achieve the surface effect with high matching degree. The simulation of cartilage thickness is completed by a compatible rod element, and the closed mechanical system is generated by the adaptive rod element at the edge of the shell structure, and no new nodes are generated between the compatible rod element and adaptive rod element, which improves the calculation efficiency. The weaving technology of the adaptive rod unit needs good mechanical insight and sensitivity [5, 19].

## 5. Conclusion

In this paper, a three-dimensional finite element model of the knee joint including main anatomical structures is established, and the transverse isotropy of ligaments is considered. Based on the finite element model and the same ligament constitutive equation, a three-dimensional finite element model of the knee joint including main anatomical structures is reconstructed by reverse modeling technology. The transverse isotropy of ligaments is considered. Based on the same constitutive model, the parameters of three different ACL mechanical experimental curves were fitted, and the mechanical properties of the knee joint under different ACL properties were compared, and the influence of different ACL mechanical curves on the finite element simulation of the knee joint was quantitatively analyzed. The effects of three different ACL mechanical property curves on the biomechanical properties of the knee joint were compared, which has good guiding significance for how to select tissue mechanical property parameters and predict possible changes in future finite element analysis. It is proved that selecting different ACL mechanical performance curves will have an impact on the results of finite element simulation. In the future, we should pay enough attention to the setting of the corresponding tissue mechanical properties of the knee joint and the construction and verification of the model.

RETRACTED

## Figures and Tables

**Figure 1:** Comparison of ACL mechanical models based on three kinds of mechanical curve fitting.

**Table 1:** Material parameters and unit types of each component.

Organization	*E* (MPa)	*μ*	Unit type
Bone	12000	0.3	SOLID92
Cartilage	12	0.46	SHELL93, LINK8
Meniscus	40	0.49	SOLID92

**Table 2:** Material parameters of the knee ligament.

	*C*_1_	*C*_2_	*C*_3_	*C*_4_	*C*_5_	*λ* ^*∗*^	*D*
PCL	3.25	0.0	0.120	87.18	431.06	1.035	0.000308
MCL	1.44	0.0	0.570	48.00	467.10	1.063	0.000347
LCL	1.44	0.0	0.570	48.00	467.10	1.063	0.000500
ACL (1)	1.00	0.0	2.59	10.31	422.27	1.268	0.000101
ACL (2)	1.24	0.0	0.869	45.11	413.95	1.056	0.000403
ACL (3)	1.95	0.0	0.0139	116.2	535.04	1.046	0.000257

**Table 3:** Comparison of knee joint displacement under 134 N femoral posterior thrust.

	Model 1	Model 2	Model 3
Back displacement of the femur (mm)	4.70	3.23	3.47
Proximal displacement of the femur (mm)	0.379	−0.0341	0.066
Outward displacement of the femur (mm)	2.54	2.00	1.83
Tibia varus (.)	1.2	1.1	1.0
Internal rotation of the tibia (?)	5.5	4.6	4.2

## Data Availability

The data used to support the findings of this study are available upon request to the author.
